# A Clinical Study on the Use of Yiqi Yangxue Decoction Combined with Chemotherapy to Promote Rapid Postoperative Recovery in Patients with Non-Small Cell Lung Cancer

**DOI:** 10.1155/2022/7073893

**Published:** 2022-09-09

**Authors:** Junyan Liang, Yue Wang, Ling Zheng, Hui Mei

**Affiliations:** Xiangyang Central Hospital, Affiliated Hospital of Hubei University of Arts and Science, Xiangyang 441000, Hubei, China

## Abstract

**Purpose:**

To observe the promotion effect of Yiqi Yangxue decoction combined with chemotherapy on the rapid recovery of non-small cell lung cancer (NSCLC) patients after surgery.

**Methods:**

Eighty postoperative NSCLC patients admitted to our hospital from April 2019 to September 2021 were divided into a chemotherapy group (*n* = 40) and a traditional Chinese medicine (TCM) group (*n* = 40) according to a random sampling method. Both groups were treated with surgery and postoperative routine chemotherapy. The TCM group was treated with Yiqi Yangxue decoction, one dose per day, starting from the first day of chemotherapy. Four weeks was a course of treatment, and three courses of treatment were taken continuously. The levels of serum tumour markers (carcinoembryonic antigen (CEA), cytokeratin 19 fragment (CYFRA21-1), carbohydrate antigen 125 (CA-125)), immune function indicators (CD3^+^, CD4^+^/CD8^+^, and NK cells), Pittsburgh Sleep Quality Index (PSQI) score, and Insomnia Severity Index (ISI) were compared between the two groups before and after treatment, and the clinical efficacy of the two groups was assessed with reference to the WHO efficacy criteria for solid tumours, and the toxic side effects of the two groups were assessed with reference to the WHO classification criteria for the toxic effects of chemotherapeutic drugs.

**Results:**

After treatment, the levels of CEA, CYFRA21-1, and CA-125 were lower than those before treatment in both groups, and they were lower in the TCM group than in the chemotherapy group (*P* < 0.05). After treatment, the levels of CD3^+^, CD4^+^/CD8^+^, and NK cells in both groups were higher than before treatment, and they were higher in the TCM group than in the chemotherapy group (*P* < 0.05). After treatment, the PSQI and ISI scores of both the groups were lower than those before treatment, and they were higher in the TCM group than in the chemotherapy group (*P* < 0.05). After treatment, the overall tumour control rate was higher in the TCM group than in the chemotherapy group (*P* < 0.05). During the treatment period, the TCM group showed lower levels of gastrointestinal reactions, leucopenia, anaemia, and neurotoxicity than the chemotherapy group (*P* < 0.05).

**Conclusion:**

The combination of Yiqi Yangxue decoction combined with chemotherapy for postoperative NSCLC patients can effectively reduce serum tumour marker levels, enhance the body's immune function and sleep quality, and the patient's efficacy and toxicity reduction are obvious, which is conducive to the rapid recovery of many indicators after surgery.

## 1. Introduction

Lung cancer is the most common malignancy in China and worldwide in terms of incidence and mortality. Non-small cell lung cancer (NSCLC) is the most common histological type of lung cancer, accounting for over 80% of lung cancer cases [1, 2]. The lack of specific clinical manifestations in the early stages of NSCLC and the insensitivity of available screening indicators have been reported, resulting in most patients developing intermediate to advanced stages by the time they are seen [3]. Although surgical resection is currently the primary treatment option, satisfactory results are not yet available and patients still need prolonged chemotherapy after surgery to fight off cancer cells. However, while killing cancer cells, chemotherapy also causes some damage to normal tissue cells, such as gastrointestinal reactions, bone marrow suppression, and other adverse reactions [4].

According to Chinese medicine, the occurrence of tumors is related to the patient's positive qi condition, and weak positive qi is one of the main causes of tumor development. As the saying goes, “When the righteousness exists within, the evil cannot dry up” and “Where the evil comes together, its qi will be deficient.” Once a tumour has formed, it can further damage the vital energy, making it even more deficient in qi, blood, yin, and yang. Chemotherapy is a poisonous attack, and although it can be used against lung cancer, it can also disturb the body's qi, deplete the body's vital energy, and damage the body's qi and blood. Yiqi Yangxue decoction is mainly used in the treatment of postpartum blood clots with pain and syncope [5, 6]. Modern research has shown that the herbal medicine Yiqi Yangxue decoction can also inhibit the progression of malignant tumours, reduce adverse effects, improve immune function, and enhance the quality of life. Based on the above, the present study was conducted to observe the effect of Yiqi Yangxue decoction with chemotherapy in promoting the rapid recovery of NSCLC patients after surgery. The report is as follows.

## 2. Materials and Methods

### 2.1. General Data

Eighty postoperative NSCLC patients admitted to our hospital from April 2019 to September 2021 were divided into a chemotherapy group (*n* = 40) and a traditional Chinese medicine (TCM) group (*n* = 40) according to a random sampling method. A comparison of the clinical characteristics of the two groups is shown in Table 1, none of which were significantly different and comparable (*P* > 0.05).

### 2.2. Inclusion Criteria

① Those who met the diagnostic criteria of the national comprehensive cancer network (NCCN) guidelines for the diagnosis and treatment of non-small cell lung cancer and are diagnosed as NSCLC by imaging and pathological examination [7]; ② patients diagnosed as stage III—IV by the TNM staging criteria [8] of NSCLC; ③ age 18∼70 years old; ④ Those who planed to undergo surgical treatment in our hospital without preoperative radiotherapy and chemotherapy; ⑤ those who had accepted the survey with good compliance and completed the assessment.

### 2.3. Exclusion Criteria

① Patients and their family members who refused surgical treatment or had chemotherapy contraindications; ② patients with tumors of other organs; ③ primary diseases with other important organs such as the heart, liver, and kidney or serious dysfunction of related organs; ④ patients with infection before operation, such as pulmonary infection and urinary system infection; ⑤ patients who had a history of hormone or immunosuppressant use or complicated with autoimmune diseases within 3 months before operation.

### 2.4. Medication Regimen

Both groups were treated with operation and routine chemotherapy after operation, while the TCM group was treated with Yiqi Yangxue decoction.

Chemotherapy regimen: Gemcitabine (Jiangsu Haosen Pharmaceutical Co., Ltd.) 100 mg/m^2^ was injected intravenously on the first day, once a week. After 3 weeks of continuous use, the drug was stopped for 1 week and then continued to be used. Cisplatin (Jiangsu Haosen Pharmaceutical Co., Ltd.) 80 mg/m^2^ was injected intravenously on the first day, once a week. After continuous use for 3 weeks, the drug was stopped for 1 week and then continued to be used. 21 days was a cycle, and the treatment lasted for 3 cycles.

Prescription of Yiqi Yangxue decoction: *Codonopsis pilosula*, *Angelica sinensis*, and Radix Paeoniae Alba each 20 g; *Astragalus membranaceus*, and Caulis Spatholobi each 30 g; Ligusticum wallichii 9 g; Licorice, Pericarpium Citri Reticulatae Viride, and Pericarpium Citri Reticulatae each 6 g. Syndrome differentiation plus or minus: For those with weak spleen qi, add 15 g each of Atractylodes Macrocephala and Poria; For those with liver stagnation and Qi stagnation, add 15 g each of Bupleurum Chinense and Radix Curcumae; For those with poor appetite, add 30 g each of Grain Sprout and Malt; For those with abdominal distension, add 9 g of Magnolia Officinalis; For those with nausea and vomiting, add 15 g of Inula. Usage: Take 300–400 ml thick decoction of various drugs, take orally twice in the morning and evening, 1 dose per day, take it on the first day of chemotherapy, 4 weeks as a course of treatment, 3 courses in a row.

### 2.5. Assessment Indicators

1. Tumour markers: before and after treatment, 5 ml of fasting elbow vein blood was collected from patients, centrifuged at 3000 r/min for 10 min, and the supernatant was stored at −80°C after completion for testing. The carcinoembryonic antigen (CEA), cytokeratin 19 fragment (CYFRA21-1) and carbohydrate antigen 125 (CA-125) were determined by chemiluminescence immunoassay. The kits were supplied from Wuhan PhD Biological Engineering Company. CEA values of 0–4.3 ng/ml is considered normal, CYFRA21-1 <3.3 ng/ml is considered normal and CA-125 < 35 U/ml is considered normal.
2. Immune function index: before and after treatment, 5 ml of fasting elbow venous blood was collected from the patient, centrifuged at 3000 r/min for 10 min, and the supernatant was stored at −80°C after completion for measurement. CD3^+^, CD4^+^, CD8^+^, and NK cell levels were measured by BD flow cytometry and the kits were supplied from Wuhan PhD Biological Engineering Company.
3. Sleep quality: before and after treatment, patients' sleep quality was assessed using the Pittsburgh Sleep Quality Index (PSQI) [9] score and the Insomnia Severity Index (ISI) [10]. The PSQI scores out of 21 and the ISI scores out of 28, both of which were inversely correlated with sleep quality.
4. Efficacy assessment: after treatment, the clinical efficacy of the two groups was assessed with reference to the WHO criteria for the efficacy of solid tumours [11]. Complete remission (CR): complete disappearance of the tumour lesion, no new lesion appears and lasts for more than 4 weeks; partial remission (PR): ≥50% shrinkage of the tumour lesion, no new lesion appears and lasts for more than 4 weeks; stable disease (SD): <50% shrinkage of the tumour lesion, ≤25% increase in size, no new lesion appears and lasts for more than 4 weeks; progressive disease (PD): >25% increase in size or new lesion appears. Overall control rate = (CR + PR)/40 × 100%.
5. Toxic side effects: during treatment, the major toxic side effects (gastrointestinal reactions, leukopenia, anaemia, and neurotoxicity) of the two groups were graded 0, I, II, III, and IV with reference to the WHO criteria for grading the toxic side effects of chemotherapeutic drugs [12].

### 2.6. Statistical Methods

SPSS 20.0 statistical software was used to analyse the data. Statistical information was described in (%) using the *χ*^2^ test and measurement information is expressed in (*x* ± *s*) using the *t*-test, with *P* < 0.05 being a statistically significant difference.

## 3. Results

### 3.1. Comparison of Serum Tumour Markers between the Two Groups

After treatment, the levels of CEA, CYFRA21-1, and CA-125 were lower than those before treatment in both groups, and they were lower in the TCM group than in the chemotherapy group (*P* < 0.05). (Figure 1).

### 3.2. Comparison of Immune Function Indicators between the Two Groups

After treatment, the levels of CD3^+^, CD4^+^/CD8^+^, and NK cells in both the groups were higher than before treatment, and they were higher in the TCM group than in the chemotherapy group (*P* < 0.05). (Figure 2).

### 3.3. Comparison of Sleep Quality between the Two Groups

After treatment, the PSQI and ISI scores of both groups were lower than those before treatment, and they were lower in the TCM group than in the chemotherapy group (*P* < 0.05). (Figure 3).

### 3.4. Comparison of Clinical Outcomes between the Two Groups

After treatment, the overall tumour control rate was higher in the TCM group than in the chemotherapy group (*P* < 0.05). (Table 2).

### 3.5. Comparison of Toxic Side Effects between the Two Groups

During the treatment period, the TCM group showed lower levels of gastrointestinal reactions, leucopenia, anaemia, and neurotoxicity than the chemotherapy group (*P* < 0.05). (Table 3).

## 4. Discussion

NSCLC belongs to the category of “lung accumulation” and “lung rock” in Chinese medicine. Mainly due to the entry of wind and cold evil into the body, causing dysfunction of the lung and spleen, patients suffer from lung qi stagnation, spleen loss of health, qi stagnation, blood stasis and phlegm, which eventually lead to NSCLC. Surgery and chemotherapeutic drugs are the main treatment for NSCLC, but while they remove the evil toxins, they will deplete the body's fluids and blood, resulting in a deficiency of positive energy, so the recurrence rate is still high after surgery, and postoperative treatment still needs to be supplemented with other drugs.

For these conditions, TCM practitioners often use medicines that benefit the Qi and nourish the blood, invigorate the blood, and remove blood stasis. In the Yiqi Yangxue decoction, *Codonopsis pilosula* and *Astragalus* membranaceus can support the body and strengthen the essence, benefit the Qi and nourish the blood, and improve the immunity of the body. Radix Paeoniae Alba has the effects of dispelling wind and dehumidification and has a regulating effect on the improvement of wind cold invasion of the body. Caulis Spatholobi can dispel wind and promote blood circulation, relax muscles and activate collaterals, and promote the recovery of the body. Licorice, Pericarpium Citri Reticulatae Viride, and Pericarpium Citri Reticulatae have antibacterial and anti-inflammatory effects, which can effectively inhibit the occurrence of postoperative inflammation and reduce postoperative tumor recurrence and metastasis. *Angelica sinensis* and Ligusticum wallichii have the function of promoting blood circulation and removing blood stasis, which can restore the normal blood circulation and promote the postoperative recovery. The combination of the above drugs has been proven by modern pharmacological studies [13] to be able to induce apoptosis of tumour cells by enhancing the activity of oxygen free radicals, inhibit the growth and proliferation of tumour cells by blocking the division phase, and enhance the immunity of the body.

Related studies [14–16] pointed out that CEA, CYFRA21-1, and CA-125 are all tumour markers, and their levels are important for the diagnosis of NSCLC disease. The CEA is an acidic glycoprotein found in the membranes of tumour cells differentiated from the fetal intestine and endodermal layers, and is present at high levels in NSCLC and positively correlates with the stage and differentiation of NSCLC metastasis. The CYFRA21-1, mainly a cytokeratin 19 fragment, is commonly found in the lung and the breast epithelium and has the highest sensitivity in squamous lung cancer with an AUC of 0.91. CA-125 is derived from coelom epithelial cells, which is usually used as a tumor marker of ovarian cancer, but its level can also be significantly increased in lung cancer, breast cancer, and colorectal cancer. This shows that all three are of great value in the pathological diagnosis and assessment of the efficacy of NSCLC. The serum CEA, CYFRA21-1, and CA-125 levels of patients in the TCM group were significantly lower than those in the chemotherapy group after treatment in this study. It indicates that chemotherapy supplemented with Yiqi Yangxue decoction treatment significantly inhibited the secretion of tumour markers and promoted postoperative recovery in patients with NSCLC after surgery.

The immune function of the body has a close relationship with the occurrence and development of tumors. When tumors occur, the body can exert antitumor effects through both cellular and humoral immunity [17]. Cellular immunity is mediated by T lymphocytes, mainly through a combination of T cells, NK cells, and macrophages in the body. CD3^+^ is a common marker on the surface of mature T cells. CD4^+^ has an auxiliary effect on the expression of T cells. CD8^+^ can inhibit T cells, inhibit the immune response of the body, and it is conducive to the formation, growth, and metastasis of tumors. NK cells have a broad-spectrum antitumor effect and can kill homologous and heterogeneous tumor cells [18]. Therefore, the detection of T cell subsets and NK cell activity in the peripheral blood of NSCLC patients has certain value for judging the immune function of tumor patients and has certain clinical significance for monitoring tumor recurrence and evaluating prognosis. The results showed that after treatment, the levels of CD3^+^, CD4^+^/CD8^+^, and NK cells in the TCM group were higher than those in the chemotherapy group. It shows that Yiqi Yangxue decoction can effectively regulate the level of peripheral blood T lymphocytes in patients with NSCLC after chemotherapy and has a positive significance in promoting the rapid recovery of immune function.

The morbidity and mortality of NSCLC increases exponentially in the elderly population over 65 years of age and, due to the complexity of the condition of elderly cancer patients, treatment options for such patients should be more focused on improving their quality of life [19, 20]. However, various toxic side effects of chemotherapy such as gastrointestinal reactions, leukopenia, anaemia, neurotoxicity, hair loss, and sleep disturbances can adversely affect the quality of life of patients [21]. The results of this study show that Yiqi Yangxue decoction not only has significant potency-boosting and toxicity-reducing functions but also significantly improves patients' sleep conditions and enhances sleep quality.

In summary, the combination of Yiqi Yangxue decoction combined with chemotherapy for postoperative NSCLC patients can effectively reduce serum tumour marker levels, enhance the body's immune function and sleep quality, and the patient's efficacy and toxicity reduction are obvious, which is conducive to the rapid recovery of many indicators after surgery.

## Figures and Tables

**Figure 1:** Comparison of serum tumour markers between the two groups. Note: compared with the chemotherapy group before treatment, ^*∗*^*P* < 0.05; compared with the TCM group before treatment and the chemotherapy group after treatment, ^*∗∗*^*P* < 0.05.

**Figure 2:** Comparison of immune function indicators between the two groups. Note: compared with the chemotherapy group before treatment, ^*∗*^*P* < 0.05; compared with the TCM group before treatment and the chemotherapy group after treatment, ^*∗∗*^*P* < 0.05.

**Figure 3:** Comparison of sleep quality between the two groups. Note: compared with the chemotherapy group before treatment, ^*∗*^*P* < 0.05; compared with the TCM group before treatment and the chemotherapy group after treatment, ^*∗∗*^*P* < 0.05.

**Table 1:** Comparison of clinical features between the two groups.

Information	Chemotherapy group (*n* = 40)	TCM (*n* = 40)	*t*/*χ*^2^	*P*
Age (years old)	53.90 ± 6.80	54.40 ± 5.16	0.370	0.712
Body mass index (kg/m^2^)	22.96 ± 2.12	22.86 ± 2.26	0.204	0.839
Male (*n*, %)	26 (65.00)	24 (60.00)	0.213	0.644
History of smoking (*n*, %)	17 (42.50)	19 (47.50)	0.202	0.653
Tumour stages (*n*, %)			0.487	0.485
III	24 (60.00)	27 (67.50)		
IV	16 (40.00)	13 (32.50)		
Pathology type (*n*, %)			0.202	0.653
Adenocarcinoma	23 (57.50)	21 (52.50)		
Squamous carcinoma	17 (42.50)	19 (47.50)		
Surgical procedure (*n*, %)			0.237	0.888
Lung lobectomy	25 (62.50)	23 (57.50)		
Pneumonectomy	12 (30.00)	14 (35.00)		
Pulmonary segment resection	3 (7.50)	3 (7.50)		

**Table 2:** Comparison of clinical outcomes between the two groups (*n*, %).

Grade	Chemotherapy group (*n* = 40)	TCM group (*n* = 40)	*χ * ^2^	*P*
CR	0 (0.00)	0 (0.00)	—	—
PR	9 (22.50)	18 (45.00)	4.528	0.033
SD	15 (37.5)	16 (40.00)	0.053	0.818
PD	16 (40.00)	6 (15.00)	6.270	0.012
Overall control rate	9 (22.50)	18 (45.00)	4.528	0.033

**Table 3:** Comparison of toxic side effects between the two groups (*n*, %).

Group	Gastrointestinal reactions	Leucopenia	Anaemia	Neurotoxicity
Chemotherapy group (*n* = 40)				

0	21 (52.50)	26 (65.00)	27 (67.5)	26 (65.00)
I	8 (20.00)	8 (20.00)	6 (15.00)	8 (20.00)
II	6 (15.00)	4 (10.00)	4 (10.00)	3 (7.50)
III	4 (10.00)	2 (5.00)	2 (5.00)	2 (5.00)
IV	1 (2.50)	0(0.00)	1 (2.50)	1 (2.50)

TCM group (*n* = 40)				

0	31 (77.50)	34 (85.00)	36 (90.00)	35 (87.50)
I	5 (12.50)	4 (10.00)	3 (7.50)	4 (10.00)
II	3 (7.50)	2 (5.00)	1 (2.50)	1 (2.50)
III	1 (2.50)	0 (0.00)	0 (0.00)	0 (0.00)
IV	0 (0.00)	0 (0.00)	0 (0.00)	0 (0.00)

## Data Availability

The data used to support the findings of this study are available at a reasonable request from the corresponding author.
